The article "Low-density lipoprotein nanomedicines: mechanisms of targeting, biology, and theranostic potential" was published in 2021. Journal: Drug Deliv.

# Low-density lipoprotein nanomedicines: mechanisms of targeting, biology, and theranostic potential

**DOI:** 10.1080/10717544.2021.1886199

**Published:** 2021-02-17

**Authors:** Lin Di, Andrei Maiseyeu

**Affiliations:** Cardiovascular Research Institute, School of Medicine, Case Western Reserve University, Clevehand, OH, USA

**Keywords:** Low-density lipoproteins, eat-me signal, oxidized lipoprotein, synthetic LDL mimics, molecular imaging, drug delivery

## Abstract

Native nanostructured lipoproteins such as low- and high-density lipoproteins (LDL and HDL) are powerful tools for the targeted delivery of drugs and imaging agents. While the cellular recognition of well-known HDL-based carriers occurs via interactions with an HDL receptor, the selective delivery and uptake of LDL particles by target cells are more complex. The most well-known mode of LDL-based delivery is via the interaction between apolipoprotein B (Apo-B) – the main protein of LDL – and the low-density lipoprotein receptor (LDLR). LDLR is expressed in the liver, adipocytes, and macrophages, and thus selectively delivers LDL carriers to these cells and tissues. Moreover, the elevated expression of LDLR in tumor cells indicates a role for LDL in the targeted delivery of chemotherapy drugs. In addition, chronic inflammation associated with hypercholesterolemia (i.e., high levels of endogenous LDL) can be abated by LDL carriers, which outcompete the deleterious oxidized LDL for uptake by macrophages. In this case, synthetic LDL nanocarriers act as ‘eat-me’ signals and exploit mechanisms of native LDL uptake for targeted drug delivery and imaging. Lastly, recent studies have shown that the delivery of LDL-based nanocarriers to macrophages via fluid-phase pinocytosis is a promising tool for atherosclerosis imaging. Hence, the present review summarizes the use of natural and synthetic LDL-based carriers for drug delivery and imaging and discusses various mechanisms of targeting.

## Introduction

Lipoproteins are naturally-occurring supramolecular particles comprised of various lipids that form complexes with specific apolipoproteins. Lipoproteins consist of a non-polar core – composed primarily of cholesteryl esters and triacylglycerides – and an amphiphilic outer shell of phospholipids and embedded cholesterols and apolipoproteins, held together by noncovalent forces (Feingold & Grunfeld, 2018). While the main function of lipoproteins is to transport insoluble lipids via blood plasma to the liver, adipocytes, and other tissues (Rensen et al., 2001; Dashty et al., 2014), recent studies have demonstrated the potent antioxidant and immunomodulatory effects of lipoproteins (Kontush et al., 2003; Yu et al., 2010; Brites et al., 2017). Lipoproteins are classified into four major types based on size, the density of the lipoprotein particle, and their functional roles: i) chylomicrons – which are composed mainly of triacylglycerols (TAGs) (80–85% w/w) and compose less than 3% of proteins – are the largest diameter (75–600 nm) and lowest density class of lipoprotein particles; ii) very low density lipoproteins (vLDLs) are 30–80 nm in diameter and are composed of TAGs (40–45% w/w), free and esterified cholesterol, and contain a core structural protein, apolipoprotein B (ApoB); iii) low density lipoproteins (LDLs) are 18–25 nm in size and are composed primarily of cholesterol and cholesteryl esters and single ApoB protein; and iv) high density lipoproteins (HDLs) – the smallest lipoprotein particle (<12 nm) – have the highest protein content (35–55% w/w) and contain the apolipoproteins ApoA1 and ApoA2 (as well as other apolipoproteins and non-apolipoproteins), phospholipids, and cholesterol, which are all are readily exchangeable (Oram & Vaughan, 2000; Cavigiolio et al., 2010; Sundaram & Yao, 2012; Mei & Atkinson, 2015).

The article "Low-density lipoprotein nanomedicines: mechanisms of targeting, biology, and theranostic potential" was published in 2021. Journal: Drug Deliv.

Although lipid and protein contents of lipoproteins can be variable depending on species (e.g. human, animal), disease state, nutrition, and genetics (John Chapman, 1986; Levy et al., 2000; German et al., 2006; Hegele, 2009; Dron & Hegele, 2016), apolipoproteins are functionally classified as either water insoluble and non-exchangeable (ApoB family) or water soluble and exchangeable (ApoA, ApoC, and ApoE families) (Babin et al., 1997; Curtiss et al., 2006; Phillips, 2013). Whereas non-exchangeable apolipoproteins remain on the same lipoprotein particle from biosynthesis to degradation, exchangeable apolipoproteins (ApoA, ApoC and ApoE families of lipoproteins) are able to interact with a number of lipid-bearing structures and molecules (e.g. vesicles, membranes, and other lipoproteins) (Jonas & Phillips, 2008). Apolipoproteins also play a role in the synthesis of LDL and HDL, as their carrier proteins (ApoB and ApoA-I, respectively) are released from the liver in a complex with nascent vLDL or from the liver and intestine as lipid-free ApoA-1, respectively. ApoB and ApoA-I subsequently recruit lipids, triglycerides, and cholesterol, which are transported between peripheral tissues and the liver as part of the functional processes called forward and reverse cholesterol transport (Tall, 1998; Huang, Elvington, et al., 2015).

In addition to structural heterogeneity, lipoproteins also differ functionally (i.e., in transporting lipids, cholesterol, and TAGS). LDL – which accounts for 80–90% of all circulating cholesterol – mainly serves to transport cholesterol from the blood to peripheral tissues, and is ultimately removed from the blood by binding to LDL receptors that are expressed in peripheral tissue cells in a process known as forward cholesterol transport (Tall, 1998). In contrast, HDL originates from the liver as nascent ApoA1, binds to ATP-binding cassette protein A1(ABCA1)/ABCG1, and transfers free, unesterified cholesterol from peripheral tissues to the liver in a process called reverse cholesterol transport (Lewis & Rader, 2005; Huang, Elvington, et al., 2015). HDL is eventually cleared from circulation by scavenger receptor B1 (SRB1), which is expressed by liver cells (Harders-Spengel, 1989; Tall, 1998). Although it was thought that SRB1 was only expressed by hepatocytes (Varban et al., 1998), our recent work demonstrates SRB1 expression in sinusoidal liver endothelial cells in a mouse model (Ganesan et al., 2016).

The article "Low-density lipoprotein nanomedicines: mechanisms of targeting, biology, and theranostic potential" was published in 2021. Journal: Drug Deliv.

Lipoprotein mimetics is a burgeoning field in which lipoproteins can be modified in a variety of ways to be used as nanocarriers in targeted drug delivery as well as in imaging (Skajaa et al., 2010; Thaxton et al., 2016). Lipoproteins make near ideal delivery agents because i) they are biocompatible and biodegradable, ii) they can be targeted to a specific receptor via apolipoproteins, iii) their cores can be loaded with drugs/imaging probes (i.e., payloads) by the reconstitution of the core, and iv) they are amenable for bioconjugation, PEGylation, and other surface modifications (Thaxton et al., 2016).

As the role of HDL-based nanocarriers have been well reviewed and investigated (Skajaa et al., 2010; McMahon et al., 2015; Kuai et al., 2016), the current review will focus on LDL-based theranostics, which have not been reviewed most recently.

The uptake of LDL occurs via receptor-mediated endocytosis by a family of structurally similar LDL receptor proteins that includes LDL receptor-related protein (LRP or megalin), very-low density lipoprotein (vLDL) receptor, and apolipoprotein E receptor-2 (ApoER2) (May et al., 2007). While it was originally thought that lipids were the only ligands bound by the LDL receptor family, it has since been shown that LRP is a scavenger receptor that binds to proteases, lipases, protease inhibitors, and exotoxin A from a bacterium (Figure 1) (Willnow et al., 1999). Therefore LRP and other members of this receptor family are involved in various biological processes unrelated to lipoprotein metabolism (Herz & Strickland, 2001).

**Figure 1.** Schematic representation of main routes of lipoprotein engulfment. (A) Under normal conditions, native, unmodified LDL has two main routes of engulfment: through its cognate receptor LDLR and via macro-/micropinocytosis. The resulting intracellular pathways of such engulfment are also distinct, producing either clathrin coated vesicles or membrane-encased LDL that may be directly released into the cytoplasm or proceed to endo-lysosomal route of degradation. (B) Modified LDL particles, including oxidatively-modified LDL (oxLDL) may also be engulfed through macro-/micropinocytosis in atherosclerosis conditions, however, their main route of cellular uptake is through scavenger receptors, thus epitomizing ‘eat-me’ type of uptake. (C) Oxidized lipids from oxLDL may be transferred to neighboring cells or engulfment of oxLDL may result in cellular apoptosis. Both of which render the uptake through scavenger and pattern recognition receptors. Interestingly, the uptake of apoptotic bodies or pathogens occurs through much similar mechanisms, and often involves milieu-oxidized intermediates.

The article "Low-density lipoprotein nanomedicines: mechanisms of targeting, biology, and theranostic potential" was published in 2021. Journal: Drug Deliv.

Under normal conditions, the receptor-mediated endocytosis of LDL occurs when ApoB-100 from LDL binds to LDLR and forms a complex embedded in clathrin-coated pits and vesicles (Figure 1) (Nykjaer & Willnow, 2002). The complex in the clathrin-coated pit subsequently separates from the cell membrane, forms a coated vesicle that depolymerizes its tubules to become an endosome, and fuses with sorting vesicles (i.e., late endosomes). During the maturation of endosomal compartments, a decrease in luminal pH (as low as pH 5) results in the dissociation of LDL from the LDLR. LDLR is then recycled back to the cell membrane, and LDL is catabolized into amino acids and free cholesterol, which is stored in the cells and in turn downregulates the expression of LDLR on the cell surface (Bareford & Swaan, 2007).

In atherosclerosis, macrophages internalize ApoB-containing lipoproteins during plaque development and convert them to cholesterol-laden foam cells, resulting in an inflammatory response that ultimately drives the pathogenesis and cardiovascular events associated with the disease (Chistiakov et al., 2016). The downregulation of LDLR early in the formation of foam cells led to the hypothesis of LDL modification and its uptake by different pathways (Brown & Goldstein, 1975; Herijgers et al., 2000). This downregulation was originally hypothesized to serve as a feedback mechanism to limit the amount of cellular cholesterol and halt foam cell formation (Brown & Goldstein, 1975). However, it is now known that increased oxidative stress in the arterial wall promotes the conversion of LDL to oxidized LDL (ox-LDL, see below in a designated chapter), which is efficiently taken up by macrophages. The ox-induced accumulation of cholesterol by macrophages results in foam cell formation and triggers damage-associated molecular patterns (DAMPs) that are recognized by the scavenger receptors (SR-A1, SR-A2, SR-B1, CD36), lectin-like oxidized LDL receptor 1 (LOX1), scavenger receptor expressed by endothelial cells 1 (SREC1), and scavenger receptor for phosphatidylserine and oxidized LDL (SR-PSOX; also known as CXCL16) (Moore & Freeman, 2006). Collectively, the pattern recognition receptors (PRRs) of macrophages recognize modified LDL as DAMPS, or an ‘eat-me’ signal (Figure 1). This molecular signal is expressed on the surface of a cell or large particle and is recognized by a corresponding receptor on a phagocyte (e.g. macrophage) to initiate selective phagocytosis of that cell (endocytosis or pinocytosis, if it is a particle). Ox-LDL binding to several scavenger receptors on macrophages appears to play a vital role in disease pathogenesis and it is thought that PRRs recognize ox-LDL as an ‘eat-me’ signal in a manner similar to ‘eat-me’ signals on oxidatively damaged/apoptotic cells. In agreement with this, Terpstra et al (Terpstra et al., 1997, 1998). showed that the binding and phagocytosis of oxidatively-damaged red blood cells or apoptotic thymocytes to mouse peritoneal macrophages were very strongly inhibited by ox-LDL but not by native LDL or acetylated LDL. These early reports on ox-LDL biology clearly established that ox-LDL induces DAMPs similarity to apoptotic cells, and are thus strong ‘eat-me’ signals for atherosclerotic plaque macrophages.

The article "Low-density lipoprotein nanomedicines: mechanisms of targeting, biology, and theranostic potential" was published in 2021. Journal: Drug Deliv.

In addition, the enzymatic modification of LDL via lipolytic enzymes such as proteases and lipases in the arterial wall resulting in the aggregation of LDL molecules, which are taken up by macrophages via micropinocytosis independently of scavenger receptors (Buono et al., 2009; Kruth, 2013). Thus, it is clear that multiple pathways could participate in the development of foam cells in atherosclerosis (Figure 1). Using these mechanisms of absorption, native LDL, ox-LDL, and LDL/ox-LDL mimics in the form of synthetic nanoparticles are able to serve as specific ‘eat-me’ signals, and are thus of great interest for their applications in drug delivery (Bagalkot et al., 2016). While the role of other lipoproteins (i.e., HDL) in drug delivery has been extensively reviewed, in-depth reviews on LDL/ox-LDL (and their ‘eat-me’ analogs) are lacking (Damiano et al., 2013; Huang, Cruz, et al., 2015). Indeed, HDL has proven useful as a vehicle for drug delivery, the main mode of delivery of this potentially antiatherogenic lipoprotein likely involves reverse cholesterol transport pathways (Duivenvoorden et al., 2014; Pérez-Medina et al., 2015; Rohatgi, 2015; Sanchez-Gaytan et al., 2015), and is thus completely different from that of LDL/ox-LDL, which can serve as an ‘eat-me’ signal that is internalized via a wide range of scavenger receptors.

‘Eat-me’ signals are imperative in all living systems and are molecular clues that drive the removal of dead/apoptotic cells in the body (Ravichandran, 2011; Morioka et al., 2019). There are several well-known cell surface molecules that serve as ‘eat-me’ signals, such as phosphatidylserine (PtdSer), calreticulin, DAMPs, and others (Bianchi, 2007; Ravichandran, 2011; Morioka et al., 2019). The role of low density lipoprotein (LDL) and oxidized LDL (ox-LDL) have also been reviewed with respect to their ‘eat-me’ signal properties (Grimsley & Ravichandran, 2003; Bagalkot et al., 2016; Tajbakhsh et al., 2018), although not that extensively. Traditionally, ‘eat-me’ signals are perceived as molecular cues that are commonly used by apoptotic cells to induce selective phagocytosis. While these signals are diverse and span a variety of structural conformational and functional moieties, they all serve to remove cell- or molecular debris. They differ greatly from ‘don’t eat-me’ signals, which serve to inhibit the ability of a cell to be engulfed by a phagocyte (Grimsley & Ravichandran, 2003; Poon et al., 2014). Specifically, it is now well established that the cells expressing high levels of CD47 inhibit phagocytic uptake through multiple mechanisms and these mechanisms were reviewed elsewhere (Oldenborg, 2004; Barclay & Van den Berg, 2014; Zhang & Huang, 2016). ‘Eat-me’ and ‘don’t eat-me’ are opposing signaling systems that cross-regulate cell and debris engulfment to play a critical role in the balance between normal physiology and pathogenesis.

The article "Low-density lipoprotein nanomedicines: mechanisms of targeting, biology, and theranostic potential" was published in 2021. Journal: Drug Deliv.

As these signals are crucial for maintaining homeostasis in biological systems, they offer a unique opportunity for targeted delivery of imaging and therapeutic agents, especially in pathologies associated with enhanced or muted phagocytic responses, such as atherosclerosis and cancer. While the biology of these signals has been extensively reviewed, this article highlights LDL/oxLDL ‘eat-me’ signals in the arena of drug delivery for imaging and therapy, i.e., theranostics. In the following chapters, this review will focus on ‘eat-me’ mechanisms of action and applications of select LDL-based theranostics.

## LDL as an ‘Eat-Me’ signal: imaging applications

### LDL nanoparticles and MRI

A significant body of work describes functional LDL-based nanoparticles for contrast enhancement in magnetic resonance imaging (MRI). In this section, we focus on native LDL nanoparticles, usually isolated from blood plasma by ultracentrifugation and subsequent modification of the surface (shell) of this lipoprotein with MRI contrast agents. We discuss the most prominent examples while providing additional references in Table 1, which also notes specific modifications of these agents and the effects observed.

The article "Low-density lipoprotein nanomedicines: mechanisms of targeting, biology, and theranostic potential" was published in 2021. Journal: Drug Deliv.

**Table 2.** Examples of reconstituted/synthetic LDL nanoparticles used in drug delivery.

Name	LDL formulation	Therapeutic payload	Disease state	Therapeutic benefit	Ref.
CSLN/ siCTGF	Reconstituted apolipoprotein-free LDLs with cationic residue outer membrane	siCTGF	Liver fibrosis	Successful targeted delivery of siRNA and dramatic improvement of patho-physiological state in liver fibrosis murine model	(Kong et al., 2013)
LDL-DHA	Reconstituted LDL loaded with docosahexaenoic acid (DHA)	DHA	Hepatocellular carcinoma murine model	Successful delivery of DHA and preferential cytotoxicity to malignant murine liver cells	(Reynolds et al., 2014)
Dox-siRNA/LDL-SCS- NPs	Reconstituted LDL loaded with both cholesterol- conjugated siRNA and doxorubicin and coupled with N-succinyl chitosan	siRNA and Dox	Hepatoma and hepatoblastoma G_2_ liver tumor models	Successful selective targeting of liver tumor cell lines and cytotoxicity of tumor cell lines with relatively low toxicity in normal cells *in vivo*	(Zhu et al., 2014)
r-SiPcBOA-LDL	Reconstituted LDL with silicon phthalocynaine oleate (SiPcBOA)	SiPcBOA	Human hepatoblastoma G2 tumor cell line	Significant increase in targeted PDT therapeutic and enhanced efficacy of PDT to tumor cell line *in vitro*	(Li et al., 2005)
r-Nc-LDL	Reconstituted LDL with silicon naphthalocynaine oleate (SiNcBOA)	SiNcBOA	Human hepatoblastoma G2 tumor line in murine model	Successful targeted tumor uptake *in vivo* with PDT potential	(Song et al., 2007)
r-Bchl-BOA-LDL	Reconstituted LDL with bacteriochlorin e6 bisoleate	Bacteriochlorin e6 bisoleate	Human hepatoblastoma G2 tumorline in murine model	Successful PDT therapeutic delivery and significant tumor regrowth delay *in vivo*	(Marotta et al., 2011)
c-Met siRNA-PEG/SLN	Reconstituted protein free LDL conjugated to PEGylated c-Met siRNA	c-Met siRNA	Glioblastoma multiforme murine model	Successful delivery of c-Met siRNA and significant attenuation of tumor growth in Glioblastoma multiforme *in vivo* model	(Jin et al., 2011)
PtSLN	Synthetic LDL mimic: PEG-conjugated solid lipid nanoparticle consisting of cholesteryl oleate and triolein as core structure lipids and DOPE, cholesterol, and DC-cholesterol as surface structure lipids with incorporation of Paclitaxel	Paclitaxel	Various lung cancer cell xenografts in murine model	Significant improvement of chemotherapeutic targeting to non-targeted Paclitaxel *in vivo*	(Kim et al., 2015)
nLDL-PO	Synthetic LDL mimic: Lipid components of phosphatidyl choline, Triolein, and cholesteryl oleate as lipid component and 18 amino acid peptide component attached to the LDL-R binding domain of ApoB-100 with incorporation of Paclitaxel oleate	Paclitaxel oleate	Glioblastoma multiforme *in vitro* study	Selective targeting and cell death of glioblastoma multiforme cells *in vitro*	(Nikanjam, Blakely, et al., 2007; Nikanjam, Gibbs, et al., 2007)
sLDL	Synthetic LDL mimic: Lipid components of phosphatidyl choline, Triolein, cholesterol, and cholesteryl oleate as lipid component and peptide mimic of ApoB-100 with incorporation of Imatinib	Imatinib	Several myeloid leukemia cell lines for *in vitro* study	Selective uptake of sLDL particle by myeloid leukemia cell lines for delivery of therapeutic	(Zhou et al., 2010)
PNP-PTX	PEG-PLA nanoparticle with conjugation of protein optimized for affinity to LDL-R (Peptide-22) and incorporation of paclitaxel	Paclitaxel	Brain glioma murine model	Enhanced BBB permeability, selective glioma targeting, and enhanced chemotherapeutic effect *in vivo*	(Zhang et al., 2013)
LDL-receptor targeted liposomal drug (in combination with statin)	Anionic pegylated liposomes composed of PEG, cholesterol, and phosphocholine, and phosphoglycerol with incorporation of doxorubicin	Dox	CNS tumor cell line *in vitro* study	Significant BBB permeability, significant targeting of vehicle to tumor cell line	(Pinzón-Daza et al., 2012)
DHA-LDL	Human LDL isolated from plasma of patients with hypercholesterolemia loaded with DHA	DHA	Cancer stem cells (CSCs) derived from human hepatocellular carcinoma (HCC) cell lines and rat model of liver cancer	70–100% killing of EpCAM^+^ CD133^−^ CSCs	(Yang et al., 2018)
DHA-LDL	Reconstituted LDL loaded with DHA	DHA	Biodistribution study in rat	Focused ultrasound facilitated LDL-DHA to cross blood–brain barrier (BBB) and DHA-LDL was delivered and metabolized by brain cells	(Mulik et al., 2016)
DHA-LDL	Reconstituted LDL loaded with DHA	DHA	ACI rats injected with rat hepatoma cell line H4IIE	80% of tumor tissue was necrotic	(Wen et al., 2016)
PTX‐siRNA/LDL‐NSC‐LA micelles	LDL was isolated from human plasma and then formed complex with siRNA	siRNA and paclitaxel	Brain metastases of triple negative breast cancer (TNBC)	Designed co-delivery system that significantly improved antitumor effects of paclitaxel by silencing the multidrug resistance gene of tumors with siRNA	(Yang et al., 2017)
pH-sensitive ApoB-100/ oleic acid-Dox/ NLC (AODN) nanoparticle	Reconstituted LDL loaded with doxorubicin bound with oleic acid which could be hydrolyzed at low pH	Dox	Breast cancer	Showed a increased accumulation at tumor site, expressed coherent pH-dependent release and effectively suppressed orthotopic breast cancer	(Li et al., 2019)
PALA-sLDL	Synthetic LDL made by lipid emulsion and lipoprotein containing LDL-R binding domain	Paclitaxel-alpha linolenic acid	U87 MG tumor-bearing mice	Reduced cytotoxicity while decreased tumor size more effectively compared to Paclitaxel alone	(Su et al., 2016)
Cholesterol-core nanoparticles (LDE)	Synthetic LDL mimic: cholesteryl oleate, phosphatidylcholine, miglyol 812 N, cholesterol, and polysorbate 80 mimic lipid component, and the LDE acquires apolipoprotein after contact with plasma	Paclitaxel	ApoE deficient mice fed with high fat diet and developed atherosclerosis	Reduced stenosis at atherosclerotic lesion area by 22%, and showed that 10–200 nm size of LDE performed similarly on therapeutic effects	(Lima et al., 2017; Freitas et al., 2018)
Cholesterol-core nanoparticles (LDE)	Synthetic LDL mimic: cholesteryl oleate, phosphatidylcholine, miglyol 812 N, cholesterol, and polysorbate 80 mimic lipid component, and the LDE acquires apolipoprotein after contact with plasma	Carmustine	New Zealand rabbits were fed a 1 % cholesterol diet for 8 weeks	Compared to control groups, the delivery system reduced lesion area by 90%	(Daminelli et al., 2016)
DHA-LDL	Human LDL isolated from patients with family hypercholesterolemia history	DHA	Human liver tumor cell lines: PLC/PRF/5 and HepG2; and rat hepatoma cell line: H4IIE	Induced both rat hepatoma and human hepatocellular carcinoma cell death through ferroptosis pathway	(Ou et al., 2017)
The amphipathic hybrid peptide decorated lipoprotein- mimic nanoparticles	Reconstituted LDL decorated with lipid-binding motif of apoB-100 and loaded with paclitaxel	Paclitaxel	Carcinoma cell lines and M109 lung tumor-bearing mice	Internalized with positive assist via folate receptor and increased antitumor efficiency of paclitaxel in M109 tumor-bearing mice	(Qian et al., 2019)
ApoE3-LDL mimic polymeric nanoparticles	LDL-mimic nanoparticles made from PEG-PCL with ApoE3 integrated on the surface	Donepezil	Human neuroblastoma (SH-SY5Y) cells and Alzheimer’s disease D induced rats	Reduced neurotoxicity *in vitro* by inhibiting Aβ oligomer formation and promoted cognitive ability in vivo	(Krishna et al., 2020)

The article "Low-density lipoprotein nanomedicines: mechanisms of targeting, biology, and theranostic potential" was published in 2021. Journal: Drug Deliv.

**Table 1.** Examples of LDL nanoparticles used in imaging.

Name	LDL formulation	Contrast agent	Imaging modality	Image enhancement	Ref.
Gd^3+^-LDL	Reconstituted LDL with intercalation of DO3A derivative with conjugation to Gd^3+^	Gd^3+^	MRI	Enhanced imaging of atherosclerotic plaque *in vivo*	(Lowell et al., 2012; Yamakoshi et al., 2011)
Gd-DTPA-SA- LDL	Reconstituted LDL with combination of DTPA-SA to serve as chelator for Gd3+	Gd^3+^	MRI	Enhanced imaging of human hepatoblastoma G2 xenografts *in vivo*	(Corbin et al., 2006)
AT101-LDL complex	Reconstituted LDL with AT101 complex	Gd-157 isotope	MRI& Boron-Neutron Capture Therapy (BNCT)	MR imaging and therapy in pulmonary lung metastasis model	(Alberti et al., 2015)
LOX-1-USPIO	USPIO conjugated to LOX-1 antibody	Iron oxide	MRI	Enrichment of LOX-1 USPIO particles in atherosclerotic lesions seen by MRI	(Wen et al., 2014)
(rITG)LDL	Reconstituted LDL with poly-iodinated triglyceride (ITG)	ITG	CT	Enhancing CT image intensity in human hepatoblastoma G2 cells *in vitro*	(Hill et al., 2010)
Au-LDL	Reconstituted LDL labeled with gold nanocrystals	Au	CT	Enhanced CT imaging at a subcellular, cellular, and anatomical level of Lewis lung carcinoma tumor models *in vivo*	(Allijn et al., 2013)
Gd-DTTA-Si- LDL	Reconstituted LDL with combination of DTTA-Si to serve as chelator for Gd3+	Gd^3+^	MRI	Enhanced imaging contrast in tumor	(Mirzaei et al., 2020)
LDL-gold	Native LDL	Gold	Transmission electron microscopy (TEM)	Identify the exact 3 D distribution of nanoparticles and clustering behavior over time in single cell	(Baudoin et al., 2013)
Gd-LDL	Reconstituted LDL with combination of DO3A	Gd^3+^ and sulfo- rhodamine	MRI and high emission fluorescent imaging	The particles selectively accumulated at atheroslerosic plaques and strongly enhanced MRI contrast in mouse model	(Fracassi et al., 2020)

The most common modification of LDL is through its lipid core, via attachment of lipophilic moieties. With this approach, the LDL remains intact, retaining its native structure. Gadolinium (Gd^3+^)-based imaging contrast agents are usually incorporated into LDL particles via intercalation of Gd-chelating lipids. For instance, Lowell et al. have developed MRI-visible LDL nanoparticles via intercalation of a long alkanoyl moiety anchoring within native LDL lipid shell, while chelating Gd^3+^ through DO3A (Yamakoshi et al., 2011; Lowell et al., 2012). The synthesis involved the stabilization with tropolone, which is particularly interesting, as tropolone is known to strongly coordinate Gd^3+^, thus significantly improving the stability of the final LDL-conjugate. This also helped to remove unbound Gd, which is important due to the high toxicity of free Gd^3+^ (Ramalho et al., 2016). The conjugate was tested in vivo in an apoE^−/−^ mouse model of atherosclerosis that showed a significant enhancement of atheroma using a 9.4 T magnet and multi-slice fast spin-echo sequences. The authors posited that the macrophages could be the cellular component responsible for the enhancement in plaque and that such a probe could serve as nonimmunogenic contrast agents for atherosclerosis (Yamakoshi et al., 2011; Lowell et al., 2012), although the immune response was not tested. Similarly, Corbin et al. incorporated amphiphilic Gd chelates into LDL and targeted them to hepatoblastoma G2 xenografts in a murine tumor model. LDL particles were isolated from fresh plasma by sequential centrifugation and Gd-carrying DTPA-SA (diethylenetriaminepentaacetic acid stearylamine) chelating lipid was incorporated directly into LDL’s lipid core (Corbin et al., 2006). The main mechanism of targeting of these functionalized LDL contrast agents to hepatic cancer cells was shown to occur through the LDLR-dependent pathway. These agents were also shown to compete with native LDL and demonstrated the absence of the uptake in ldlA7 cells (LDL receptor-deficient cells) (Corbin et al., 2006). This early report is a nice proof-of-concept demonstrating the ability of LDL-based carriers to target tumors, as it is well-known that many tumor cells upregulate LDL transporters and receptors (Menrad & Anderer, 1991; Li et al., 2004). In line with this, Alberti et al. suggested a theranostic approach to imaging and treatment of lung cancer via Boron Neutron Capture Therapy (BNCT) (Alberti et al., 2015). This methodology relies on the use of LDL particles as a vehicle for dual boron/Gd agent based on a carborane unit bearing ten boron atoms and an aliphatic chain that facilitates the binding of LDL particles. Boron neutron capture therapy-based cancer treatment works on the principle of boron load delivery by such LDL carrier homing to cancer tissue and followed by exposure to a beam of irradiated neutrons. In the target tissue, the LDL carrier reacts with boron-10 that captures the slow-moving neutron to form boron-11, while releasing charged alpha particles and gamma rays – lethal to cancer cells. Such an approach was hypothesized to be particularly useful for pulmonary metastases where surgical resection is challenging. Indeed, when administered in the mouse model of lung metastasis, MR signal enhancement was observed both in tumor and liver, and while BNCT treatment retarded tumor growth in the first 25 days after irradiation, slow regrowth was noted after one month. This could be attributed to low LDLR expression in the lung and, therefore, suboptimal delivery.

The article "Low-density lipoprotein nanomedicines: mechanisms of targeting, biology, and theranostic potential" was published in 2021. Journal: Drug Deliv.

Another particularly interesting example that demonstrates a potential for oxLDL targeted agents, is a nanoparticulate carrier that targets LOX-1, an oxLDL receptor (Wen et al., 2014). Pathological Ox-LDL formation is linked to highly oxidative conditions in the vessel wall during the development of atherosclerotic lesions (Boullier et al., 2001). Accumulation of ox-LDL in macrophages and other immune cells within the vessel wall results in the release of inflammatory cytokines that triggers the underlying endothelial cells to produce a variety of adhesion factors and pro-inflammatory molecules, thus amplifying cardiovascular inflammation (Mohty et al., 2008; Duewell et al., 2010). The overexpression of oxLDL receptor LOX-1 is known to stimulate various signaling pathways leading to endothelial dysfunction and plaque destabilization (Xu et al., 2013). Intriguingly, pathological LOX-1 overexpression can be taken advantage of by utilizing the LOX-1-directed targeting mechanism. Thus, ultrasmall superparamagnetic iron oxide (UPSIO) nanoparticles coated with an antibody specific to LOX-1 selectively targeted carotid atherosclerotic lesions in apoE^−/−^ mice (Wen et al., 2014). The results showed clear contrast enhancement of the LOX-1-expressing plaques using T2 MRI imaging 8 h after injection, with some particles persisting in the circulation up to 24 h. Apart from targeting carotid lesions this study further showed that LOX-1-targeted-UPSIO could be used as a potential noninvasive imaging method of LOX-1-related glomerular disease, where increased expression of LOX-1 plays an important pathogenic role. Therefore, LOX-1 targeting is an attractive avenue that can be exploited for LDL/oxLDL delivery to pathologies where the overexpression of this receptor plays a detrimental role (see below for a separate chapter on oxLDL targeting).

### LDL nanoparticles and CT

Targeted molecular probes enhance specificity and binding to tissue enabling contrast enhancement for cancer/cardiovascular imaging. LDL-based nanoparticles offer key advantages of biocompatibility and receptor-mediated targeting mechanism via LDLR that was explored in multiple studies using computed tomography (CT) imaging (Table 1). In one study, LDL nanoparticles loaded with a CT contrast poly-iodinated triglyceride (ITG) selectively targeted cultured human hepatoblastoma G2 (HepG2) cells that overexpress LDLR (Hill et al., 2010). Here, lyophilized LDL was extracted with an organic solvent (heptane) for subsequent reconstitution with ITG. Such reconstituted LDL-ITG was dissolved in an aqueous buffer to yield rLDL-ITG nanoparticles with an effective iodine loading of 0.78 mg/mL. Importantly, reconstitution did not alter the targeting functionality of LDL, and the CT imaging of HepG2 cells showed significant contrast enhancement over control cells. It is clear that LDL core loading with dyes/imaging probes affords targeted molecular imaging agents, however, it may also offer important insights on biomolecular interactions through various imaging methodologies, especially when performed simultaneously. For example, Fayad and colleagues demonstrated that LDL particles can be labeled with gold nanocrystals (Au-LDL), which retain the native LDL structure, provide contrast enhancement in CT and fluorescence imaging, but also offer the ability to deliver therapeutically active gold nanocrystals (Allijn et al., 2013). Strong uptake in cells expressing high levels of LDLR (HepG2 hepatocytes, J774A.1 macrophages and B16-F10 melanoma) was noted and the uptake was competitively inhibited by co-incubation with native LDL, suggesting an LDLR-mediated interaction of Au-HDL with cellular LDLR. *In vivo,* when Au-HDL was administered in low-density lipoprotein receptor knockout (LDLR KO), the biodistribution studies showed 50% lower liver uptake vs. wild type mice. This study also showed that when Au-HDL was administered in B16-F10 tumor-bearing mice and imaged by CT, Au-HDL accumulated in tumor-associated macrophages (TAMs), highly expressing LDLR. The results from this study and the work of others indicate that loading of LDL with organic dyes, metals (Au), or inorganic molecules (quantum dots) do alter the physicochemical nature and targeting of LDL. This is particularly exciting as such an approach paves the way for the development of targeted CT contrast agents as well as for studying LDL interactions in atherosclerotic plaques *in vivo*. Additional examples of LDL-based CT contrast agents and their properties are presented in Table 1.

The article "Low-density lipoprotein nanomedicines: mechanisms of targeting, biology, and theranostic potential" was published in 2021. Journal: Drug Deliv.

## LDL as an ‘eat me signal’: therapeutic applications

### Reconstituted LDL and drug delivery

In addition to the aforementioned advantages of LDL-based nanoparticles in their ease of synthesis using a reconstitution (extraction of native biological material from blood plasma LDL followed by re-formation of the LDL particle in the presence of synthetic entity), their intrinsic targeting ability is of great potential (Table 2). Native LDL’s main protein component is apolipoprotein B100 (apoB100) provides stability and maintains the precise size and structure of reconstituted LDL nanoparticles, but most importantly, allows for targeted binding to the LDLR. This affords selective uptake of LDL carriers by themselves, unlike other synthetic lipidic nanoparticles such as micelles, liposomes, and even semi-synthetic exosomes, which must possess a separate targeting mechanism for selective uptake. LDL carriers and mimics utilize the endocytic and pinocytic absorption mechanisms inherent to endogenous LDL and are metabolized in liver hepatocytes, making reconstituted LDL particles ideally suited for drug delivery and imaging of hepatic tissue. Additionally, as mentioned above, some cancers overexpress LDLR and can be targeted via their tumor-associated macrophages.

The article "Low-density lipoprotein nanomedicines: mechanisms of targeting, biology, and theranostic potential" was published in 2021. Journal: Drug Deliv.

This intrinsic targeting capability of LDL can be taken advantage of through conjugation strategies to a standalone nanocarrier if reconstitution of LDL does not allow for sufficient payload. A particularly interesting example of such a strategy is a study by Zhu et al. that reports a hybrid polymeric nanoparticle assembled from native LDL particles covalently attached to succinyl-chitosan nanoparticles. Interestingly, the covalent reaction through the amine groups on LDL via carbodiimide chemistry allowed for facile coupling of succinyl chitosan. Such coupling allowed for a hybrid ‘two-in-one’ construct where the LDL was loaded with *mdr1* siRNA while chitosan nanoparticles were conjugated with doxorubicin (Dox). The goal of the study was to deliver siRNA to silence the multidrug-resistant gene in tumors simultaneously with chemotherapy (Zhu et al., 2014). The study demonstrates that both Dox and siRNA are released into the cytoplasm upon uptake by liver cells. Gene silencing *in vitro* was observed with a reduction in *mdr1* gene expression at 48 h in HepG2 cells, although non-LDL cholesterol-modified siRNA also showed a similar effect, which authors attributed to the presence of lipophilic cholesterol that could interact with the cell membrane for efficient uptake. The tumor-targeting capability of chitosan-LDL nanoparticles was evaluated by near-infrared fluorescence imaging after injection of nanoparticles in three types of liver tumor models: mice bearing H22 tumor *in situ*, subcutaneously transplanted HepG2 tumor, and HepG2 tumor *in situ ‒* all showed nanoparticle accumulation in liver tumor indicating proof-of-concept targeting. Interestingly, these nanoparticles were cleared via renal filtration as seen by strong fluorescence signals in the kidneys post 24 h. Unfortunately, the study does not report on gene silencing effects *in vivo,* although this approach seems to be an effective strategy to deliver both cytotoxic drugs and gene silencing therapy to tumors.

Due to the affinity of LDL’s lipophilic core, lipidic therapeutics are near ideal for LDL reconstitution. Thus, Reynolds et al. examined the ability of native LDL to deliver polyunsaturated omega-3 fatty acid (PUFA) docosahexaenoic acid (DHA) as an anticancer agent against hepatocellular carcinoma in a murine model (Reynolds et al., 2014). All PUFAs are highly lipophilic fats and therefore are challenging to deliver intravenously as free molecules as they can aggregate in the bloodstream, endangering the patient with potential emboli formation. Remarkably, LDL particles that naturally have a high lipid to protein ratio can accommodate large payloads of PUFA in their core. Reconstituted LDL-DHA particles were found to contain 1453 molecules of DHA per LDL and were quasi spherical-shaped with an average particle diameter of 18.3 ± 0.53 nm, which is very similar to native unmodified LDL. Circular dichroism spectrophotometry demonstrated that the secondary structure of apo-B100 in LDL-DHA was very similar to that of native LDL, but a 37% reduction in apo-B100 protein content was noted. This did not impact the stability of the conjugate which remained unchanged for almost one month at room temperature. The mechanism of antitumor efficacy of LDL-DHA was due to induction of reactive oxygen species (ROS), likely through mitochondrial metabolism activation by DHA (Ng et al., 2005). In malignant TIB-75 hepatocyte-like cell line LDL-DHA were more efficacious as compared to its counterpart TIB-73 normal hepatocytes. The selective oxidative damage in TIB-75 malignant hepatocyte cells was hypothesized to be due to higher basal levels of oxidative stress present in these tumor cells.

The article "Low-density lipoprotein nanomedicines: mechanisms of targeting, biology, and theranostic potential" was published in 2021. Journal: Drug Deliv.

Non-pharmacological cancer treatments such as photothermal and photodynamic therapies are gaining momentum with the field of nanomedicine advancing toward imaging-based monitoring of responsiveness to treatment. Photothermal nanotherapy uses metal nanoparticles such as gold nanoparticles irradiated with near-infrared light that is when adsorbed increases the local tissue temperature and thus preferentially killing the cancer cells. Photodynamic (PDT) nanotherapy uses a photosensitizer molecule that absorbs the irradiated light and converts it to vibrational energy (heat) that causes toxicity to the cancer cells. Although research has advanced on the preclinical side, safety issues in the clinic still remain a concern and thus are under active investigation. Thus, Li and Song et al. examined the delivery of (Nc) naphthalocyanine-reconstituted and phthalocyanine-reconstituted LDL nanoparticles as PDT payloads to humans hepatoblastoma G2 (HepG2) tumor cells (Li et al., 2005; Song et al., 2007). In these studies, Nc was synthetically modified to bear neutral and hydrophobic SiNcBOA, tetra-*t*-butyl silicon naphthalocyanine bisoleate, for efficient anchorage into LDL lipid core. Importantly, this modification prevents Nc aggregation/stacking as observed with other planar aromatic structures and increases Nc’s photosensitizing ability. The tumor-targeting efficacy was studied by spectrophotometry that showed significant absorption enhancement in tumor tissue versus muscle (8:1) 2 h post-injection. Additional experiments showed that the targeting was through the LDLR endocytic pathway (Figure 1). Similarly, Marotta et al. demonstrated that a reconstituted bacteriochlorin e6 bisoleate low-density lipoprotein (r-Bchl-BOA-LDL) could be irradiated at a longer wavelength of 748 nm than usual, and was shown to serve as an adequate photosensitizer in PDT. The application of r-Bchl-BOA-LDL in the murine model significantly delayed tumor regrowth in mice bearing HepG2 tumors (Marotta et al., 2011). The above studies establish LDL as a significant targeting apparatus for PDT agents in various cancers.

The article "Low-density lipoprotein nanomedicines: mechanisms of targeting, biology, and theranostic potential" was published in 2021. Journal: Drug Deliv.

### Synthetic LDL mimics and drug delivery

In contrast to reconstituted LDL that retains the native structure of LDL with intact ApoB-100 protein, synthetic LDL particles are assembled from commercial phospholipids but lack ApoB-100 protein (Table 2). For example, solid lipid nanoparticles synthesized from synthetic lipids with the same composition as that of LDL and a targeting ligand (epidermal growth factor receptor (EGFR)-targeting antibody) chemically conjugated to the surface of LDL have been reported as drug delivery vehicles for highly hydrophobic insoluble paclitaxel (Kim et al., 2015). The lipids included cholesteryl oleate, triolein as the core structure lipids and cholesterol, DC-cholesterol as the surface structure lipids. Paclitaxel was loaded at the reconstitution step yielding synthetic LDL-drug encapsulated nanoparticles. A similar approach was used to load LDL-like lipids with short interfering RNA (siRNA) and immobilize them onto cationic solid lipid nanoparticles (CSLNs). These possessed the same outer and inner lipid composition as that of native LDL in an effort to target connective tissue growth factor with corresponding siRNA (siCTGF) as a potential liver fibrosis therapy (Kong et al., 2013). The resulting CLSNs had a diameter in the range of 106.2 ± 5.4 nm, which is approximately 5 times higher than native LDL (18–25 nm). *In vitro* studies in HepG2 cells demonstrated that a FAM-labeled CLSN-siRNA fluorescent complex showed effective endosomal escape and nuclear localization. In the hepatic fibrosis rat model, administered CLSN-CTGF-siRNA demonstrated high liver biodistribution after a single intravenous injection and showed significant improvement in liver function, manifesting in the decrease of circulating liver enzymes alanine transaminase (ALT), aspartate transaminase (AST), total bilirubin (TBIL), and total albumin (ALB). Serum cytokines (IL-6, TNF-α, TGF-β) and CTGF levels themselves (by western blot) were reduced as compared to CLSN without targeting siRNA. Immunohistochemistry for liver fibrosis showed no signs of collagen deposition.

In a series of very intriguing studies, Nikanjam et al. developed a synthetic LDL mimic as a drug delivery vehicle for glioblastoma multiforme (Nikanjam, Blakely, et al., 2007; Nikanjam, Gibbs, et al., 2007). This nanoparticle contained a peptide constructed with both a lipid-binding motif and the ApoB-100 LDLR binding domain. This synthetic LDL mimic served as a vehicle for delivery of paclitaxel oleate in the core of the particle, termed nano-LDL containing paclitaxel oleate (nLDL-PO) (Nikanjam, Blakely, et al., 2007; Nikanjam, Gibbs, et al., 2007). The results showed cell death in the glioblastoma multiforme cell line, consistent with the hypothesis of higher uptake of LDL particles in these LDLR-expressing glioblastoma cell. A more extensive in vivo study would be of particular interest because of natural ability of LDL to cross the blood–brain barrier (BBB) (Dehouck et al., 1997), a bottleneck for many glioblastoma therapies (van Tellingen et al., 2015; Arvanitis et al., 2020).

The article "Low-density lipoprotein nanomedicines: mechanisms of targeting, biology, and theranostic potential" was published in 2021. Journal: Drug Deliv.

In settings of chronic myeloid leukemia (CML), Zhou et al. examined the potential for drug delivery to CML progenitor cells via a synthetic LDL nanoparticle (sLDL) (Zhou et al., 2010). This study showed significant targeted uptake of the sLDL, providing a possible drug vehicle for imatinib, a CML therapeutic drug, to enhance the eradication of CML progenitor cells. Further research has shown targeted drug delivery to the LDLR by incorporating a specific protein with high affinity to the LDLR, a peptide-22, into a biocompatible poly(ethylene glycol)-poly(lactic acid) (PEG-PLA) nanoparticle. These PEG-PLA loaded with paclitaxel transported the payload of paclitaxel across the BBB and targeted glioma cells via LDLR (Zhang et al., 2013). As mentioned above, LDL vectors are particularly exciting in their ability to cross the BBB (Xu et al., 2015), to realize their translational potential for brain delivery, extensive follow-up studies are warranted.

Of special interest are approaches that are designed to regulate LDLR expression simultaneously with delivery via LDL carriers. Such a strategy may enable facilitated uptake of LDL carriers, especially if modulation of LDLR expression is site-specific. In one of the earlier attempts to achieve this, Pinzón-Daza et al. demonstrated a proof-of-principle by incorporating Dox in an anionic nanoparticle that mimics LDL (decorated with an ApoB-100 peptide that binds to LDLR), while simultaneously administering a statin (mevastatin or simvastatin) to upregulate the expression of the LDLR in cells in an *in vitro* transwell-type of the assay (Pinzón-Daza et al., 2012). Authors propose that such a ‘Trojan Horse approach’ may have many applications in drug delivery to various CNS diseases in which traversing the BBB is an obstacle. However, robust experiments in animal models are needed to demonstrate the specificity of such an approach, like statins, if delivered off-target, may inadvertently redirect the LDL carriers to sites of highest LDLR expression (e.g. liver).

The article "Low-density lipoprotein nanomedicines: mechanisms of targeting, biology, and theranostic potential" was published in 2021. Journal: Drug Deliv.

Interestingly, neuronal cells that express LDLR on their cell surface are able to accept polymeric nanoparticles via LDLR-mediated uptake, as shown by Hasadsri et al. (2009). Polybutylcyanoacrylate (PBCA) nanoparticles incorporating small protein, GTPase rhoG were absorbed by cultured neurons, *in vitro* and their uptake was inhibited by blocking LDLR (Hasadsri et al., 2009).

Another fascinating example is an LDL carrier designed to alleviate glioblastoma invasiveness. Thus, the siRNA-mediated targeting of c-MET, a protein was shown to mediate tumor invasiveness in glioblastoma multiforme, was accomplished through cationic solid lipid nanoparticle formed from reconstituted LDL and complexed with pegylated-cMet-siRNA. Such particles, referred to as CLSN-Peg-cMet-siRNA, showed significant tumor regression in a murine model of glioblastoma multiforme. This study by Jin et.al. is an important advancement in the field, because of demonstrated in vivo efficacy of LDL carriers to cross BBB – one of the most challenging endeavors in brain tumor drug delivery (Jin et al., 2011).

### OxLDL and its therapeutic potential

During the onset of atherosclerosis, the altered blood flow at arterial branches causes disturbances in the endothelial cell layer. The disrupted endothelium becomes permeable to circulating LDL and extracellular matrix (ECM) proteins that accumulate in the arterial walls and undergo various modifications. One of the most important modifications is the oxidation of accumulated LDL resulting in the formation of oxLDL (Boullier et al., 2001). The formed oxLDL is antigenic and inflammatory and its accumulation within the arterial wall stimulates the endothelial cells resulting in the secretion of proinflammatory chemokines, including CC-chemokine ligand 5 (CCL5) and CXC-chemokine ligand 1 (CXCL1) (Zhou et al., 2011). Endothelial adhesion factors (ICAM-1, VCAM-1) along with chemokines aid in the recruitment and adhesion of monocytes in the arterial wall with a subsequent differentiation to plaque macrophages (Kuznetsova et al., 2020). Resident plaque macrophages recognize oxLDL as a strong ‘eat-me’ signal and thus internalize oxLDL via macropinocytosis or scavenger receptor-mediated pathways resulting in foam cell build-up (Moore & Freeman, 2006). Another major factor for the uptake of oxLDL by scavenger receptors is their high negative charge due to oxidation, which reduces their affinity to LDLR and increases their affinity for scavenger receptors (Ohki et al., 2005). Due to the importance and high prevalence of oxLDL-dependent mechanisms of uptake in atherosclerosis, oxLDL mimetics or oxLDL-like carriers are thus particularly interesting for their use in atherosclerosis.

The article "Low-density lipoprotein nanomedicines: mechanisms of targeting, biology, and theranostic potential" was published in 2021. Journal: Drug Deliv.

Similar to LDL-mimicking nanoparticles that adopt LDLR pathway to deliver therapeutic and imaging agents, scavenger receptors can be targeted, as reported in a paradigm-shifting discovery of a library of amphiphilic sugar-based molecules (AMs). AMs mimic the charge and hydrophobicity of oxLDL and are able to bind scavenger receptors with high affinity. The initial discovery by Uhrich et al. reported sugar-based amphiphilic polymers that were composed of short hydrophobic segment (alkyl chain) on mucic acid conjugated to hydrophilic PEG segment that spontaneously can assemble into oxLDL-mimicking micelles (Tian et al., 2004). In subsequent studies, the same group of authors identified the exact structural features of the AMs that contributes to the enhanced binding to scavenger receptor (Iverson et al., 2010). A lead molecule was also identified that was shown to block oxLDL uptake by THP-1 human macrophages and mouse peritoneal macrophage cells (Chnari et al., 2006; Iverson et al., 2010). Further, the authors found that if the negative charge was increased on the hydrophobic portion of the molecule or if the PEG architecture was changed, it did not affect the ability of AMs to inhibit oxLDL binding. This suggests that AMs could further be modified for serum stability without affecting their ability to block oxLDL uptake (Hehir et al., 2012). The binding affinity of AMs can be enhanced by tweaking various parameters of the backbone, making AMs even more versatile carriers. Thus, when the backbone was modified with L-tartaric acid conjugation, the binding affinity significantly increased as compared to the parent AM molecule, M12P5, indicating that stereochemistry among other factors is an important contributor in AM binding (Poree et al., 2013). Similarly, to achieve better *in vivo* and serum stability Lewis and Moghe et al. reported the incorporation of AM micelles in nanoparticles and using a library screening approach to identify serum-stable AMs (Lewis et al., 2015). This approach also protected AM micelles against circulating esterases. Interestingly, AM-nanoparticles were assembled using a flash nanoprecipitation, a rapid mixing strategy of solvent-anti-solvent, originally developed by Robert Prud’Homme for the synthesis of polymeric assemblies (Johnson & Prud’homme, 2003). The driving force of flash nanoprecipitation is critical micelle concentration formation resulting in ‘kinetically-frozen’ stable assemblies. Using a jet mixer AM-based NP1 micelles were formed in the size of 150–200 nm, which were stable for up to 4 weeks when stored at 37 °C in buffer or for 24 h in 20% serum. NP1 showed significant binding to scavenger receptors MSR1 and CD36 in human monocyte-derived macrophages (HMDMs). Interestingly, NP1 also effectively downregulated the expression of these receptors. The significance of these results is that NP1 blocking of oxLDL binding and scavenger receptor gene downregulation would prevent uptake of oxLDL and foam cell formation resulting in atheroprotective effects *in vivo* (Petersen et al., 2014; Lewis et al., 2015). Indeed, when tested in atherosclerotic mice, the NP1 treatment caused a reduction in plaque lesion area, diminished lipid accumulation, and lowered expression of COX-1, an inflammatory marker, thus demonstrating an overall reduction in plaque inflammation. Clearly, AM and their nanoprecipitates are innovative oxLDL-mimicking carriers, however, their long-term efficacy and detailed mechanism of action need further evaluation. Additional contemporary studies of reconstituted/synthetic LDL-based delivery and therapeutic applications are presented in Table 2 (J. Yang et al., 2018; Mulik et al., 2016; Wen et al., 2016; Yang et al., 2017; Li et al., 2019; Daminelli et al., 2016; Ou et al., 2017; Qian et al., 2019; Krishna et al., 2020).

The article "Low-density lipoprotein nanomedicines: mechanisms of targeting, biology, and theranostic potential" was published in 2021. Journal: Drug Deliv.

## Conclusion

### Broadening the scope of LDL-based carriers for targeting: closing remarks

Carriers based on native LDL have vast applications for drug delivery and imaging contrast enhancement in multiple disease states. As a drug carrier LDL is a near-ideal choice since it is biocompatible and biodegradable and its targeting capability is restricted to LDL receptor-positive cells, thus increasing specificity of delivery. LDL has the potential to be modified to target receptors other than the traditional LDLR, thus ‘rerouting’ the delivery, such as by conjugation to various targeting vectors (e.g. folic acid) (Zheng et al., 2005; Chen et al., 2007), much like traditional nanoparticles. This, unfortunately, complicates the overall design of the carrier, posing the question of whether the choice of LDL platform is justified. Extensive synthetic modifications often change LDL composition or/and its size (Kong et al., 2013), resulting in particles that only remotely resemble natural LDL. Many investigators posit low immunogenicity of the LDL carriers, however, in the majority of the reports these claims are unfounded due to a lack of appropriate testing. This is especially important, as with any biologic material, and particularly with LDL, as it has the intrinsic ability to be modified *in vivo* through oxidation, aggregation, enzymatic alteration, and other routes. As a matter of fact, adjuvant-vaccination approaches are currently being actively developed against oxLDL and apoB-carrying lipoproteins in atherosclerosis (Kobiyama et al., 2018, 2019). Such strategies are based on the premise that modified LDL molecules are highly immunogenic and able to activate pathogenic autoreactive CD4^+^ T-helper cells (Wolf et al., 2020).

The article "Low-density lipoprotein nanomedicines: mechanisms of targeting, biology, and theranostic potential" was published in 2021. Journal: Drug Deliv.

In the context of atherosclerotic disease, there are numerous reports on LDL particles carrying anti-inflammatory therapies delivered to foam cells and macrophages. These studies hypothesize that such delivery is a therapeutically viable strategy because foam cells/macrophages are the main target for LDL uptake and are major contributors to atherosclerotic plaque formation. Although the classic view of macrophage-derived foam cells is that they secrete pro-inflammatory molecules and escalate the inflammatory cascade in atherosclerosis, recent research indicates that this may not be entirely the case. It was convincingly demonstrated that ‘non-foamy’ rather than ‘foamy’ macrophages are the main drivers of inflammation, at least in murine models of the atherosclerotic disease (Kim et al., 2018).

The most important (at least in these authors’ opinion) feature of LDL carriers is their ability to cross BBB and target LDLR-positive tumors as well as sub-population of neurons. This seemed like an underdeveloped area, especially given the immense importance of potential biomedical applications. Indeed, brain tumors are the most difficult to treat and neurological diseases are the world's largest cause of disability – both are likely to be addressed by LDL carriers’ LDLR-targeting mechanism. Such studies are urgently warranted in the settings of translational research.
